The article "Global Stability Analysis and Parameter Estimation for a Diphtheria Model: A Case Study of an Epidemic in Rohingya Refugee Camp in Bangladesh" was published in 2022. Journal: Comput Math Methods Med.

# Global Stability Analysis and Parameter Estimation for a Diphtheria Model: A Case Study of an Epidemic in Rohingya Refugee Camp in Bangladesh

**DOI:** 10.1155/2022/6545179

**Published:** 2022-01-27

**Authors:** Zahurul Islam, Shohel Ahmed, M. M. Rahman, M. F. Karim, M. R. Amin

**Affiliations:** ^1^Department of Mathematics, Bangladesh University of Engineering and Technology, Dhaka 1000, Bangladesh; ^2^Department of Mathematical and Physical Sciences, East West University, Dhaka, Bangladesh

## Abstract

In this article, we have developed a deterministic Susceptible-Latent-Infectious-Recovered (SLIR) model for diphtheria outbreaks. Here, we have studied a case of the diphtheria outbreak in the Rohingya refugee camp in Bangladesh to trace the disease dynamics and find out the peak value of the infection. Both analytical and numerical investigations have been performed on the model to find several remarkable behaviors like the positive and bounded solution, basic reproductive ratio, and equilibria such as disease extinction equilibrium and disease persistence equilibrium which are characterized depending on the basic reproductive ratio and global stability of the model using Lyapunov function for both equilibria. Parameter estimation has been performed to determine the values of the parameter from the daily case data using numerical technique and determined the value of the basic reproductive number for the outbreak as *ℛ*_0_ = 5.86.

## 1. Introduction

Diphtheria is a rapidly spreading disease which is generated by *Corynebacterium diphtheriae*. Diphtheria transmits in the populations, usually through respiratory droplets, like coughing or sneezing [1, 2]. When the bacteria release the poison or toxin into the body, then the actual disease appears. Fever and throat bruises are the initial symptoms of diphtheria. Besides, a thick grey layer induces the “croup,” which can block the airway and cause a barking cough. Anyone can be infected by diphtheria, but 5-7-aged children who did not receive the appropriate vaccine are usually infected [3–6]. During 1990-1995, above cases 140,000 and 4000 mortalities have been recorded worldwide through the Regional Office of World Health Organization (WHO) for Europe [7–9]. Nowadays, diphtheria is a rare outbreak in the developed world. However, in 2017, several diphtheria outbreaks occurred in Yemen and refugee camps in Bangladesh [10, 11]. In the Rohingya refugee camp in Cox's Bazar, Bangladesh, a massive-scale diphtheria pestilence was reported. Until December 26, 2017, there were an aggregate number of 2,526 cases and 27 mortalities [12]. There are diphtheria antitoxins in diphtheria treatments to stop poisons from the bacteria and antitoxins to kill the bacteria. The best way to repel diphtheria is through vaccinations [3, 4, 13]. The three shots of the diphtheria-tetanus-pertussis (DTP) vaccine were applied in massive levels to children to control the diphtheria outbreak. To break the transmission chains of the diphtheria outbreak in the Rohingya refugee camp in Bangladesh, emergency vaccination has been applied to children since December 12, 2017, and at the end of 2017, above 90% overall coverage [12].

Many researchers have studied epidemic or pandemic disease using mathematical techniques such as Wu and Zhao [14] who have mathematically analyzed an age-structured epidemic model of HIV/AIDS with HAART and spatial diffusion. In a discrete-time SIVS model with saturation incidence rate, Parsamanesh and Erfanian [15] investigated the stability and bifurcations. To examine the impact of an environmental toxin on the spread of infectious illnesses in the population, Saha and Samanta [16] used a toxin-dependent dynamical model. In a discrete time epidemic model including vaccination and vital dynamics, Parsamanesh et al. [17] investigated the stability and bifurcations. Kabir et al. [18] have analyzed the effect of border enforcement measures and socioeconomic cost in export-importation epidemic dynamics using game theory. In a random environment, Samanta and Bera [19] looked at a dynamical model of Chlamydia illness with changing total population size, bilinear incidence rate, and pulse vaccination approach. Parsamanesh and Erfanian [20] looked at the global dynamics of a model with a standard incidence rate and immunization approach. Shahrear et al. [21] have predicted and mathematically analyzed the COVID-19 outbreak in Bangladeshi scenario, and Maugeri et al. [22] have analyzed the transmission of the COVID-19 pandemic in Saudi Arabia and Indonesia. By eliciting behavioural reactions in the community, Saha et al. [23] explored an epidemic model of the COVID-19 outbreak. Liu and Zhang [24] have analyzed global stability for a tuberculosis model. Gao and Huang [25] have investigated a tuberculosis model with optimal control.

Some of the researchers have also analyzed the diphtheria epidemic, such as Vitek and Wharton [26] who have studied the potential of the reemergence of diphtheria and other vaccine-preventable infections. Zakikhany and Efstratiou [27] analyzed the current problems and new challenges of diphtheria in Europe. Torrea et al. [28] have studied the diphtheria outbreak with the SIRM model. Ilahi and Widiana [29] have developed an SEIR model for the diphtheria outbreak and analyze vaccination's effectiveness against the outbreak. Matsuyama et al. [30] have analyzed the sensitivity and ambiguity based on the basic reproductive ratio *ℛ*_0_ of the diphtheria epidemic in the Rohingya refugee camp in Bangladesh.

Due to the vulnerability of diphtheria epidemics in a confined area, we propose a controlled Susceptible-Latent-Infectious-Recovered (SLIR) model, which is an extension of the simple Susceptible-Infectious-Recovered (SIR) model by adjoining a compartment (L) that tracks the latent people in the cohort. Analytical analysis of the proposed model is performed to prove the existence, uniqueness, positivity, and bounds of the solution. Equilibria of the system and the basic reproductive ratio are also evaluated, and the global stability of the model is proven depending on the basic reproductive ratio. To illustrate the disease dynamics, parameter values are estimated from the daily case data of the outbreak in the Rohingya refugee camp in Bangladesh and found to be the equilibria of the system.

## 2. Mathematical Model

In this section, a mathematical model [31] is developed for the expanse of diphtheria into the populations, which is shown diagrammatically in Figure 1. The entire population at time *t* is indicated by *N*(*t*) that is partitioned into four groups: susceptible (*S*(*t*)), latent (asymptotic) stage (*L*(*t*)), individual affected by diphtheria in the acutely infected stage (*I*(*t*)), and recovered individuals affected by diphtheria (*R*(*t*)); here, we suppose that the recovered people are not further contagious. Here, *λ* is a constant that signifies all recruitment that enters the susceptible class, and *μ* is the natural mortality rate that leaves all classes. The infectious state has an extra mortality rate due to diseases by *α*, and *δ* is that rate in which latent infection in people becomes an acute infection. Thus, the people move to state *I* from state *L* at a rate of *δL*. Infectious people are successfully treated with a fixed rate *γ*, listing to the recovered state. Susceptible people acquire diphtheria infection among active diphtheria at rate *βSI*, where *β* signifies the infection transmission coefficient. Moreover,*l*signifies a fraction of susceptible people that earn diphtheria infection and migrate to the latent diphtheria state(*L*), at rate*lβSI*, and the residual portion,(1 − *l*), departs to the active diphtheria state(*I*). Here, the individuals of the latent class are assumed not to transmit infection.

Assembling all the aforenamed suppositions, the model concerning the transmission dynamics of diphtheria is presented by the subsequent system of differential equations:

(1) $$\begin{array}{c} \left\{\begin{array}{c} \frac{dS\left(t\right)}{dt}=\lambda -\beta S\left(t\right)I\left(t\right)-\mu S\left(t\right),\\ \frac{dL\left(t\right)}{dt}=l\beta S\left(t\right)I\left(t\right)-\left(\mu +\delta \right)L\left(t\right),\\ \frac{dI\left(t\right)}{dt}=\left(1-l\right)\beta S\left(t\right)I\left(t\right)+\delta L\left(t\right)-\left(\mu +\gamma +\alpha \right)I\left(t\right),\\ \frac{dR\left(t\right)}{dt}=\gamma I\left(t\right)-\mu R\left(t\right),\\ N\left(t\right)=S\left(t\right)+L\left(t\right)+I\left(t\right)+R\left(t\right), \end{array}\right. \end{array}$$

with following subsidiary conditions:

(2) $$\begin{array}{c} S\left(0\right)=S_{0}>0, \end{array}$$

(3) $$\begin{array}{c} L\left(0\right)=L_{0}\geq 0, \end{array}$$

(4) $$\begin{array}{c} I\left(0\right)=I_{0}\geq 0, \end{array}$$

(5) $$\begin{array}{c} R\left(0\right)=R_{0}\geq 0. \end{array}$$

## 3. Some Basic Characteristic of the Model

To retain the model's biological efficacy, we want to show the existence, positivity, and boundedness of the solutions to the differential equations for all time.

**Theorem 1 (existence of unique solution).**

Suppose that *S*_0_, *L*_0_, *I*_0_, *R*_0_ ∈ ℝ. Then, there exists continuous differentiable functions {*S*, *L*, *I*, *R* : [0, *t*_0_)⟶ℝ} for positive time (*t*_0_ > 0) such that the 4-tuple (*S*, *L*, *I*, *R*) covers (1) and (*S*, *L*, *I*, *R*)(0) = (*S*_0_, *L*_0_, *I*_0_, *R*_0_).

**Proof of Theorem 1.**

By Picard-Lindelöf theorem, it is narrated that the initial value problem **y**′(*t*) = **g**(**y**(*t*)), **y**(*t*_0_) = **y**_0_ has a unique solution **y**(*t*) for locally Lipschitz and continuous function **g** in time *t* ∈ [*t*_0_ − *ϵ*, *t*_0_ + *ϵ*], where *ϵ* > 0. As the system (1) is autonomous, it is enough to prove that the function **g** : ℝ^4^⟶ℝ^4^ is locally Lipschitz in **y**. Here, **g** is defined as

(6) $$\begin{array}{c} g\left(y\right)=\left(\begin{array}{c} \lambda -\beta SI-\mu S\\ l\beta SI-\left(\mu +\delta \right)L\\ \left(1-l\right)\beta SI+\delta L-\left(\mu +\gamma +\alpha \right)I\\ \gamma I-\mu R \end{array}\right). \end{array}$$

The Jacobian matrix of **g** is obtained as

(7) $$\begin{array}{c} \nabla g\left(y\right)=\left(\begin{array}{cccc} -\beta I-\mu & 0 & -\beta S & 0\\ l\beta I & -\left(\mu +\delta \right) & l\beta S & 0\\ \left(1-l\right)\beta I & \delta & \left(1-l\right)\beta S-\left(\mu +\gamma +\alpha \right) & 0\\ 0 & 0 & \gamma & -\mu \end{array}\right). \end{array}$$

This Jacobian is linear in ℝ^4^. Thus, ∇**g**(**y**) satisfies the continuity and differentiability for an interval *I* ∈ ℝ^4^. According to the mean value theorem,

(8) $$\begin{array}{c} \frac{\left|g\left(y_{1}\right)-g\left(y_{2}\right)\right|}{\left|y_{1}-y_{2}\right|}\leq \left|\nabla g\left(y^{*}\right)\right|, \end{array}$$

where **y**^∗^ ∈ *I*_1_. By assuming |∇**g**(**y**^∗^)| = *M*, we obtain |**g**(**y**_1_) − **g**(**y**_2_)| ≤ *M*|**y**_1_ − **y**_2_| for **y**_1_, **y**_2_ ∈ *I*_1_ and thus, **g**(**y**) is bounded locally for each **y** ∈ ℝ^4^. Therefore, for all compact subset of ℝ^4^, the derivative of **g** is continuous and bounded and thus, **g** is locally Lipschitz. Hence, according to the Picard-Lindelöf theorem, the initial value problem *y*′(*t*) = *g*(y(*t*)), *y*(0) = *y*_0_ for *t*_0_ > 0 has a unique solution *y*(*t*).

**Theorem 2 .**

The proposed model (1) is invariant in the nonnegative orthant ℝ_+_^4^.

**Proof**

Let *Y* = (*S*, *L*, *I*, *R*)^*T*^; then, model (1) will take the form

(9) $$\begin{array}{c} \frac{dY\left(t\right)}{dt}=LY+C, \end{array}$$

where

(10) $$\begin{array}{c} L=\left(\begin{array}{cccc} -\left(\beta I\left(t\right)+\mu \right) & 0 & 0 & 0\\ l\beta I\left(t\right) & -\left(\mu +\delta \right) & 0 & 0\\ \left(1-l\right)\beta I\left(t\right) & \delta & -\left(\mu +\gamma +\alpha \right) & 0\\ 0 & 0 & \gamma & -\mu \end{array}\right), \end{array}$$

and

(11) $$\begin{array}{c} C=\left(\begin{array}{c} \lambda \\ 0\\ 0\\ 0 \end{array}\right). \end{array}$$

Here, *C* ≥ 0 and in matrix L, all off-diagonal elements are greater than or equal zero. Hence, L is a Metzler matrix and the system (1) is positive invariant in ℝ_+_^4^ [32].

**Theorem 3 .**

For *t* > 0, any solution (*S*, *L*, *I*, *R*) of the model (1) with condition (2) is positive.

**Proof**

The R.H.S. of the model (1) is differentiable; therefore, connecting it with Cauchy problem covenants that there exists a unique maximal solution. The solution of the first equation of system (1) can be figured out alternatively as

(12) $$\begin{array}{c} \frac{dS\left(t\right)}{dt}+\left(\beta I\left(t\right)+\mu \right)S\left(t\right)=\lambda . \end{array}$$

The solution of Equation (12) is

(13) $$\begin{array}{c} S\left(t\right)=S_{0}e^{\left\{-\left(\mu t+\int_{0}^{t}\;\beta I\left(x\right)dx\right)\right\}}+e^{\left\{-\left(\mu t+\int_{0}^{t}\;\beta I\left(x\right)dx\right)\right\}}\times \int_{0}^{t}\;\lambda e^{\left\{\mu y+\int_{0}^{t}\;\beta I\left(u\right)du\right\}}dy, \end{array}$$

for all *t* > 0. Hence, the R.H.S. of Equation (13) is greater than or equal to zero, i.e., *S*(*t*) > 0 for all *t* > 0. In the same way, the solution of the second, third, and fourth equations of model (1) is of the form

(14) $$\begin{array}{c} L\left(t\right)=L_{0}e^{\left\{-\left(\mu +\delta \right)t\right\}}+e^{\left\{-\left(\mu +\delta \right)t\right\}}\times \int_{0}^{t}\;l\beta S\left(y\right)I\left(y\right)\;e^{\left\{\left(\mu +\delta \right)y\right\}}dy,\\ I\left(t\right)=I_{0}e^{\left\{-\left(\left(\mu +\gamma +\alpha \right)t-\int_{0}^{t}\;\left(1-l\right)\beta S\left(x\right)dx\right)\right\}}+e^{\left\{-\left(\left(\mu +\gamma +\alpha \right)t-\int_{0}^{t}\;\left(1-l\right)\beta S\left(x\right)dx\right)\right\}}\times \int_{0}^{t}\;\delta L\left(y\right)\;e^{\left\{\left(\mu +\gamma +\alpha \right)y-\int_{0}^{t}\;\left(1-l\right)\beta S\left(u\right)du\right\}}dy,\\ R\left(t\right)=R_{0}\;e^{\left\{-\mu t\right\}}+e^{\left\{-\mu t\right\}}\times \int_{0}^{t}\;\gamma I\left(y\right)\;e^{\left\{\mu y\right\}}dy, \end{array}$$

respectively. Those solutions show that all *L*(*t*), *I*(*t*), and *R*(*t*) are greater than or equal zero ∀*t* > 0.

**Theorem 4 (boundedness).**

Suppose the model (1) satisfies *S*_0_ > 0, *L*_0_ > 0, *I*_0_ > 0, and *R*_0_ > 0 and has a unique solution on [0, *t*_0_] for some *t*_0_ > 0 by Theorem 1; then, the state functions *S*(*t*), *L*(*t*), *I*(*t*), and *R*(*t*) will be bounded and be positive ∀*t* ∈ [0, *t*_0_].

**Proof**

Initially, suppose that the values of *S*(*t*), *L*(*t*), *I*(*t*), and *R*(*t*) are positive. From Theorem 1, for *t* > 0, there exists a solution on [0, *t*]. Now, denote the largest time by *𝒯*^∗^ at which all the populations are positive, or

(15) $$\begin{array}{c} T^{*}=\sup\left\{t>0:S\left(s\right),L\left(s\right),I\left(s\right),R\left(s\right)>0,\;\forall s\in \left[0,t\right]\right\}. \end{array}$$

Since all initial conditions are nonnegative and the solutions are continuous, hence, the solutions must be positive on an interval which is denoted as *𝒯*^∗^ > 0. Therefore, we calculate each term on [0, *𝒯*^∗^]: instantly, the lower bounds on *L*, *I*, and *R* can be placed.

(16) $$\begin{array}{c} \frac{dL\left(t\right)}{dt}=l\beta S\left(t\right)I\left(t\right)-\left(\mu +\delta \right)L\left(t\right)\geq -\left(\mu +\delta \right)L\left(t\right), \end{array}$$

as the reduction expressions are linear; this achieves

(17) $$\begin{array}{c} \frac{dL\left(t\right)}{L\left(t\right)}\geq -\left(\mu +\delta \right)dt, \end{array}$$

or

(18) $$\begin{array}{c} \ln\left(L\left(t\right)\right)+\ln C\geq -\left(\mu +\delta \right)t, \end{array}$$

or

(19) $$\begin{array}{c} L\left(t\right)\geq Ce^{-\left(\mu +\delta \right)t}. \end{array}$$

Applying initial condition, we get

(20) $$\begin{array}{c} L\left(0\right)\geq C,\\ \Rightarrow L\left(t\right)\geq L\left(0\right)e^{-\left(\mu +\delta \right)t}>0, \end{array}$$

for *t* ∈ [0, *𝒯*^∗^].

Again,

(21) $$\begin{array}{c} \frac{dI\left(t\right)}{dt}=\left(1-l\right)\beta S\left(t\right)I\left(t\right)+\delta L\left(t\right)-\left(\mu +\gamma +\alpha \right)I\left(t\right)\geq -\left(\mu +\gamma +\alpha \right)I\left(t\right), \end{array}$$

as the reduction expressions are linear; this achieves

(22) $$\begin{array}{c} I\left(t\right)\geq I\left(0\right)e^{-\left(\mu +\gamma +\alpha \right)t}>0,\\ \forall t\in \left[0,T^{*}\right]. \end{array}$$

Further,

(23) $$\begin{array}{c} \frac{dR\left(t\right)}{dt}=\gamma I\left(t\right)-\mu R\left(t\right)\geq -\mu R\left(t\right), \end{array}$$

i.e.,

(24) $$\begin{array}{c} R\left(t\right)\geq R\left(0\right)e^{-\mu t}>0,\\ \forall t\in \left[0,T^{*}\right]. \end{array}$$

Similarly, by placing the upper bound on *dS*/*dt*, we get

(25) $$\begin{array}{c} \frac{dS\left(t\right)}{dt}=\lambda -\beta S\left(t\right)I\left(t\right)-\mu S\left(t\right)\leq \lambda , \end{array}$$

i.e.,

(26) $$\begin{array}{c} S\left(t\right)\leq S\left(0\right)+\lambda t\leq C\left(1+t\right), \end{array}$$

where *C* is an arbitrary constant which is depending on the upper bound of *S*(0) and *λ*. Now, by adding the equations for*L*, *I*, and*R*and placing the bounds on this sum and by the positivity of these functions, for the upper bound of*S*(*t*), we get

(27) $$\begin{array}{c} \frac{d}{dt}\left(L+I+R\right)=\beta S\left(t\right)I\left(t\right)-\mu L\left(t\right)-\left(\mu +\alpha \right)I\left(t\right)-\mu R\left(t\right)\leq \beta C\left(1+t\right)I\left(t\right)+\mu L\left(t\right)+\left(\mu +\alpha \right)I\left(t\right)+\mu R\left(t\right)\leq C_{1}\left(1+t\right)\left(L+I+R\right), \end{array}$$

where *C*_1_ ≥ max{*βC*, *μ*, (*μ* + *α*)}, i.e.,

(28) $$\begin{array}{c} \left(L+I+R\right)\left(t\right)\leq C_{2}e^{t^{2}}, \end{array}$$

where the constant *C*_2_ > 0 for *t* ∈ [0, *𝒯*^∗^] that only depends on *L*(0), *I*(0), *R*(0), and *C*_1_. For the positivity of *L*(*t*), *I*(*t*), and *R*(*t*) are positive, an upper bound can be placed on both *L*, *I*, and *R* by

(29) $$\begin{array}{c} C_{2}e^{t^{2}}\geq \left(L+I+R\right)\left(t\right)\geq L\left(t\right),\\ C_{2}e^{t^{2}}\geq \left(L+I+R\right)\left(t\right)\geq I\left(t\right),\\ C_{2}e^{t^{2}}\geq \left(L+I+R\right)\left(t\right)\geq R\left(t\right). \end{array}$$

Now, *S*(*t*) can be bounded from below using

(30) $$\begin{array}{c} \frac{dS}{dt}=\lambda -\beta SI-\mu S\geq -\beta SI-\mu S\geq -\mu S-\beta C_{2}e^{t^{2}}S,\geq -C_{3}\left(1+e^{t^{2}}\right)S, \end{array}$$

where *C*_3_ ≥ max{*βC*_2_, *μ*}, ⇒(*dS*/*dt*) + *C*_3_(1 + *e*^*t*^2^^)*S* ≥ 0, i.e.,

(31) $$\begin{array}{c} S\left(t\right)\geq S\left(0\right)e^{-C_{3}\int_{0}^{t}\;\left(1+e^{\kappa^{2}}d\kappa \right)}>0. \end{array}$$

Therefore, *S*, *L*, *I*, and *R* remain rigorously positive ∀*t* ∈ [0, *𝒯*^∗^]. Hence, there exists a *t* > *𝒯*^∗^ for the continuity, at which the state variables *S*(*t*), *L*(*t*), *I*(*t*), and *R*(*t*) are still positive, which contradicts with the definition of *𝒯*^∗^ and specifies that *S*(*t*), *L*(*t*), *I*(*t*), and *R*(*t*) are rigorously positive on the whole interval [0, *t*]. Moreover, all functions remain bounded with this interval; thus, the existing interval can be further extended. Actually, the bounds on *S*, *L*, *I*, and *R* obtained earlier exist on each compact time interval. For the extension of the time interval to [0, *t*]∀*t* > 0 at which the solution endures and of the above discussion, the solutions continue both positive and bounded on [0, *t*].

## 4. Equilibria of the System

In this section, we trace the presence of steady states for the dynamical system of nonlinear ODEs (1), describing the Diphtheria disease dynamics. These steady states can be obtained by placing the R.H.S. of (1) to zero; we obtain

(32) $$\begin{array}{c} \lambda -\beta SI-\mu S=0, \end{array}$$

(33) $$\begin{array}{c} l\beta SI-\left(\mu +\delta \right)L=0, \end{array}$$

(34) $$\begin{array}{c} \left(1-l\right)\beta SI+\delta L-\left(\mu +\gamma +\alpha \right)I=0, \end{array}$$

(35) $$\begin{array}{c} \gamma I-\mu R=0. \end{array}$$

Moreover, by solving the above equations, we have found two biologically meaningful equilibrium points. We can classify these two points to be while the infection is either terminated from populations, i.e.,*L* = *I* = *R* = 0, or insists in the populations(*L* ≠ 0, *I* ≠ 0, *R* ≠ 0)as*t*grows large.

We start to determine the equilibria from the nonlinear intercommunicated terms into Equations (33), (34), and (35) that give

(36) $$\begin{array}{c} I\left(\left(1-l\right)\left(\mu +\delta \right)\beta S+\delta l\beta S-\left(\mu +\delta \right)\left(\mu +\gamma +\alpha \right)\right)=0. \end{array}$$

Thus, either *I* = 0 or *S* = (*μ* + *δ*) (*μ* + *γ* + *α*)/((1 − *l*)*μ* + *δ*)*β*. Using *I* = 0 in Equations (33), (34), and (35), we get the disease extinction equilibrium point as

(37) $$\begin{array}{c} E^{0}=\left(S^{0},L^{0},I^{0},R^{0}\right)=\left(\frac{\lambda }{\mu },0,0,0\right). \end{array}$$

By setting *S* = (*μ* + *δ*)(*μ* + *γ* + *α*)/((1 − *l*)*μ* + *δ*)*β* into Equations (32) and (35) yields the infectious persistence equilibrium that exists at the point

(38) $$\begin{array}{c} E^{*}=\left(S,L,I,R\right)=\left(\frac{\left(\mu +\delta \right)\left(\mu +\gamma +\alpha \right)}{\left(\left(1-l\right)\mu +\delta \right)\beta },\frac{l\lambda }{\left(\mu +\delta \right)}-\frac{l\mu \left(\mu +\gamma +\alpha \right)}{\beta \left(\delta +\left(1-l\right)\mu \right)},\frac{\lambda \left(\delta +\left(1-l\right)\mu \right)}{\left(\mu +\delta \right)\left(\mu +\gamma +\alpha \right)}-\frac{\mu }{\beta },\frac{\gamma \lambda \left(\delta +\left(1-l\right)\mu \right)}{\mu \left(\mu +\delta \right)\left(\mu +\gamma +\alpha \right)}-\frac{\gamma }{\beta }\right). \end{array}$$

In the biological sense, *E*^0^ is defined as a disease extinction equilibrium point in which an infection survives for a short time and then is naturally dispelled from the populations. The infection is not insisted. The other case, in which the system incline towards *E*^∗^, denoted that the populations are impotent to remove the disease spontaneously. If it closes up this remaining fact, then after a particular period, the diphtheria disease model fails its pertinency as it gets broader to keep up the populations.

## 5. Basic Reproductive Ratio

The basic reproductive ratio is also called basic reproductive rate or basic reproduction number and is denoted by *ℛ*_0_. It is a significant threshold value generated in epidemiology to mathematically identify the doubt of an infectious disease. This quantity represents the average number of infected persons generated by one infected person introduced into an entirely uninfected susceptible population. We use the next-generation method [33, 34] to obtain the basic reproductive ratio *ℛ*_0_.

Using the next-generation matrix method on the model (1), we get

(39) $$\begin{array}{c} F=\left(\begin{array}{cc} 0 & l\beta S^{0}\\ 0 & \left(1-l\right)\beta S^{0} \end{array}\right),\\ V=\left(\begin{array}{cc} \mu +\delta & 0\\ -\delta & \mu +\gamma +\alpha \end{array}\right). \end{array}$$

Therefore, we have,

(40) $$\begin{array}{c} FV^{-1}=\left(\begin{array}{cc} \frac{l\delta \beta S^{0}}{\left(\mu +\gamma +\alpha \right)\left(\mu +\delta \right)} & \frac{l\beta S^{0}}{\left(\mu +\gamma +\alpha \right)}\\ \frac{\left(1-l\right)\delta \beta S^{0}}{\left(\mu +\gamma +\alpha \right)\left(\mu +\delta \right)} & \frac{\left(1-l\right)\beta S^{0}}{\left(\mu +\gamma +\alpha \right)\left(\mu +\delta \right)} \end{array}\right). \end{array}$$

Thus, the spectral radius of the matrix*ℱ𝒱*^−1^and the basic reproductive ratio*ℛ*_0_are obtained [35].

(41) $$\begin{array}{c} R_{0}=\frac{\beta \left(\delta +\mu -l\mu \right)S^{0}}{\left(\alpha +\gamma +\mu \right)\left(\delta +\mu \right)}. \end{array}$$

Putting *S*^0^ = *λ*/*μ*, we obtain,

(42) $$\begin{array}{c} R_{0}=\frac{\lambda \beta \left(\delta +\left(1-l\right)\mu \right)}{\mu \left(\alpha +\gamma +\mu \right)\left(\delta +\mu \right)}. \end{array}$$

This expression of *ℛ*_0_ represents the basic reproductive ratio for the model (1).

**Remark 1 .**

The infectious equilibrium point with the expression of basic reproduction number *ℛ*_0_

(43) $$\begin{array}{c} \left(S^{*},L^{*},I^{*},R^{*}\right)=\left\{\frac{\lambda }{\mu R_{0}},\frac{l\lambda \left(R_{0}-1\right)}{\left(\mu +\delta \right)R_{0}},\frac{\mu }{\beta }\left(R_{0}-1\right),\frac{\gamma }{\beta }\left(R_{0}-1\right)\right\}. \end{array}$$

## 6. Global Stability Analysis

### 6.1. Global Stability at Infectious Extinction Equilibrium

For disease extinction equilibrium *E*^0^ = (*S*^0^, *L*^0^, *I*^0^, *R*^0^) = (*λ*/*μ*, 0, 0, 0), we assume the following Lyapunov function:

(44) $$\begin{array}{c} U\left(t\right)=S^{0}\left[\frac{S\left(t\right)}{S^{0}}-1-\ln\left(\frac{S\left(t\right)}{S^{0}}\right)\right]+\frac{\delta }{\left(1-l\right)\mu +\delta }L\left(t\right)+\frac{\mu +\delta }{\left(1-l\right)\mu +\delta }I\left(t\right). \end{array}$$

By differentiation, we get

(45) $$\begin{array}{c} \frac{dU}{dt}=\left(1-\frac{S^{0}}{S}\right)S^{\prime }+\frac{\delta }{\left(1-l\right)\mu +\delta }L^{\prime }+\frac{\mu +\delta }{\left(1-l\right)\mu +\delta }I^{\prime }. \end{array}$$

Substituting the values of *S*′, *L*′, and *I*′ in the above equation, we have

(46) $$\begin{array}{c} \frac{dU}{dt}=\left(1-\frac{S^{0}}{S}\right)\left[\lambda -\beta SI-\mu S\right]+\frac{\delta }{\left(1-l\right)\mu +\delta }\left[l\beta SI-\left(\mu +\delta \right)L\right]+\frac{\mu +\delta }{\left(1-l\right)\mu +\delta }\left[\left(1-l\right)\beta SI+\delta L-\left(\mu +\gamma +\alpha \right)I\right]=\left(\lambda -\mu S\right)\left(1-\frac{S^{0}}{S}\right)+\beta S^{0}I-\frac{\left(\mu +\delta \right)\left(\mu +\gamma +\alpha \right)}{\mu \left(1-l\right)+\delta }I. \end{array}$$

After substituting the value of *S*^0^ = *λ*/*μ*, we are left with

(47) $$\begin{array}{c} \frac{dU}{dt}=-\frac{{\left(\lambda -\mu S\right)}^{2}}{\mu S}+\frac{\left(\mu +\delta \right)\left(\mu +\gamma +\alpha \right)}{\mu \left(1-l\right)+\delta }\left(R_{0}-1\right). \end{array}$$

At the disease extinction equilibrium *E*^0^, the basic reproductive ratio *R*_0_ ≤ 1, and for all positive values of *S*, *L*, *I*, and *R*, it is clear that *dU*/*dt* ≤ 0. Hence, using LaSalle's Invariance Principle [36], it is concluded that the model (1) is globally asymptotically stable.

**Lemma 1 .**

The infectious extinction equilibrium (*E*^0^) of the model (1) is globally asymptotically stable when *ℛ*_0_ ≤ 1, and the disease is naturally dispelled from the populations.

### 6.2. Global Stability at Infectious Persistence Equilibrium

Since none of the state variables are zero at the infectious persistence equilibrium *E*^∗^ = (*S*^∗^, *L*^∗^, *I*^∗^, *R*^∗^), thus a Lyapunov function is assumed as

(48) $$\begin{array}{c} U\left(t\right)=\left(S-S^{*}-S^{*}\ln\left(\frac{S}{S^{*}}\right)\right)+B_{1}\left(L-L^{*}-L^{*}\ln\left(\frac{L}{L^{*}}\right)\right)+B_{2}\left(I-I^{*}-I^{*}\ln\left(\frac{I}{I^{*}}\right)\right)+B_{3}\left(R-R^{*}-R^{*}\ln\left(\frac{R}{R^{*}}\right)\right), \end{array}$$

where *B*_1_, *B*_2_, and *B*_3_ are all nonnegative constants to be obtained. This kind of Lyapunov function has been studied in [37–40].

The infectious persistence equilibrium *E*^∗^ = (*S*^∗^, *L*^∗^, *I*^∗^, *R*^∗^) satisfies the following equations:

(49) $$\begin{array}{c} \lambda =\beta S^{*}I^{*}+\mu S^{*}, \end{array}$$

(50) $$\begin{array}{c} \left(\mu +\delta \right)L^{*}=l\beta S^{*}I^{*}, \end{array}$$

(51) $$\begin{array}{c} \left(\mu +\gamma +\alpha \right)=\left(1-l\right)\beta S^{*}I^{*}+\delta L^{*}, \end{array}$$

(52) $$\begin{array}{c} \mu R^{*}=\gamma I^{*}. \end{array}$$

Now, differentiate *U* with respect to time *t*,

(53) $$\begin{array}{c} U^{\prime }=\left(1-\frac{S^{*}}{S}\right)S^{\prime }+B_{1}\left(1-\frac{L^{*}}{L}\right)L^{\prime }+B_{2}\left(1-\frac{I^{*}}{I}\right)I^{\prime }+B_{3}\left(1-\frac{R^{*}}{R}\right)R^{\prime }=\left(1-\frac{S^{*}}{S}\right)\left[\beta S^{*}I^{*}+\mu S^{*}-\beta SI-\mu S\right]+B_{1}\left(1-\frac{L^{*}}{L}\right)l\beta SI-B_{1}\left(\mu +\delta \right)L+B_{1}\left(\mu +\delta \right)L^{*}+B_{2}\left(1-\frac{I^{*}}{I}\right)\left[\left(1-l\right)\beta SI+\delta L\right]-B_{2}\left(\mu +\gamma +\alpha \right)I+B_{2}\left(\mu +\gamma +\alpha \right)I^{*}+B_{3}\left(1-\frac{R^{*}}{R}\right)\gamma I-B_{3}\mu R+B_{3}\mu R^{*}, \end{array}$$

which can be further simplified to

(54) $$\begin{array}{c} U^{\prime }=-\mu \frac{{\left(S-S^{*}\right)}^{2}}{S}+\beta S^{*}I^{*}\left(1-\frac{S^{*}}{S}\right)+SI\left[-\beta +B_{1}l\beta +B_{2}\left(1-l\right)\beta \right]+I\left[-B_{2}\left(\mu +\gamma +\alpha \right)+B_{3}\gamma +\beta S^{*}\right]+L\left[-B_{1}\left(\mu +\delta \right)+B_{2}\delta \right]+R\left[-B_{3}\mu \right]-B_{1}l\beta SI\frac{L^{*}}{L}+B_{1}l\beta S^{*}I^{*}-B_{2}\left(1-l\right)\beta SI^{*}-B_{2}\delta L\frac{I^{*}}{I}+B_{2}\left(1-l\right)\beta S^{*}I^{*}+B_{2}\delta L^{*}-B_{3}\gamma I\frac{R^{*}}{R}+B_{3}\gamma I^{*}. \end{array}$$

For the positive constants *B*_1_, *B*_2_, and *B*_3_, the coefficients of *SI*, *I*, *L*, and *R* must be zero, that is,

(55) $$\begin{array}{c} -\beta +B_{1}l\beta +B_{2}\left(1-l\right)\beta =0, \end{array}$$

(56) $$\begin{array}{c} -B_{2}\left(\mu +\gamma +\alpha \right)+B_{3}\gamma +\beta S^{*}=0, \end{array}$$

(57) $$\begin{array}{c} -B_{1}\left(\mu +\delta \right)+B_{2}\delta =0, \end{array}$$

(58) $$\begin{array}{c} -B_{3}\mu =0. \end{array}$$

By solving, the above equation (55) yields

(59) $$\begin{array}{c} B_{1}=\frac{\delta }{\mu +\delta }B_{2},\\ B_{2}=\frac{\mu +\delta }{\left(1-l\right)\mu +\delta },\\ B_{3}=0. \end{array}$$

For advantage, we set up new variables *x* = *S*/*S*^∗^, *y* = *L*/*L*^∗^, *z* = *I*/*I*^∗^, and *u* = *R*/*R*^∗^ to seek *S*, *L*, *I*, and *R* and setting the expressions of *B*_1_, *B*_2_, and *B*_3_ in Equation (54), we have

(60) $$\begin{array}{c} U^{\prime }=-\mu \frac{{\left(S-S^{*}\right)}^{2}}{S}+B_{2}\left(1-l\right)\beta S^{*}I^{*}\left(2-\frac{1}{x}-x\right)+B_{1}l\beta S^{*}I^{*}\left(2-\frac{1}{x}-\frac{xz}{y}\right)+B_{2}\delta L^{*}\left(1-\frac{y}{z}\right)+B_{3}\gamma I^{*}\left(1-\frac{z}{u}\right). \end{array}$$

Multiplying by *B*_1_ to the 2^nd^ equation of (49) and the 3^rd^ equation of (55) by *L*^∗^ yields

(61) $$\begin{array}{c} B_{1}\left(\mu +\delta \right)L^{*}=B_{1}l\beta S^{*}I^{*},\\ B_{1}\left(\mu +\delta \right)L^{*}=B_{2}\delta L^{*}. \end{array}$$

Hence, it follows that

(62) $$\begin{array}{c} -B_{1}l\beta S^{*}I^{*}+B_{2}\delta L^{*}=0. \end{array}$$

Multiplying by*F*_1_(*X*)to the last equation, where*F*_1_(*X*)is considered as a general function that will be determined later and*X* = (*x*, *y*, *z*, *u*), yields

(63) $$\begin{array}{c} -B_{1}l\beta S^{*}I^{*}F_{1}\left(X\right)+B_{2}\delta L^{*}F_{1}\left(X\right)=0 \end{array}$$

Multiplying the 4^th^ equation of (49) by *B*_3_ and the 4^th^ equation of (55) by *R*^∗^ yields

(64) $$\begin{array}{c} B_{3}\mu R^{*}=B_{3}\gamma I^{*},\\ B_{3}\mu R^{*}=0. \end{array}$$

Hence, it follows that

(65) $$\begin{array}{c} B_{3}\gamma I^{*}=0. \end{array}$$

Multiplying by*F*_2_(*X*)to the last equation, where*F*_2_(*X*)is considered as a general function that will be determined later and*X* = (*x*, *y*, *z*, *u*), yields

(66) $$\begin{array}{c} B_{3}\gamma I^{*}F_{2}\left(X\right)=0. \end{array}$$

From (54) using (63) and (66) yields

(67) $$\begin{array}{c} U^{\prime }=-\mu \frac{{\left(S-S^{*}\right)}^{2}}{S}+B_{2}\left(1-l\right)\beta S^{*}I^{*}\left(2-\frac{1}{x}-x\right)+B_{1}l\beta S^{*}I^{*}\left(2-\frac{1}{x}-\frac{xz}{y}-F_{1}\left(X\right)\right)+B_{2}\delta L^{*}\left(1-\frac{y}{z}+F_{1}\left(X\right)\right)+B_{3}\gamma I^{*}\left(1-\frac{z}{u}+F_{2}\left(X\right)\right). \end{array}$$

Now, the functions *F*_1_(*X*) and *F*_2_(*X*) are taken so that the coefficients of *L*^∗^ and *I*^∗^ are zero. For these cases, we get

(68) $$\begin{array}{c} F_{1}\left(X\right)=\frac{y}{z}-1, \end{array}$$

and

(69) $$\begin{array}{c} F_{2}\left(X\right)=\frac{z}{u}-1. \end{array}$$

Then, Equation (67) becomes

(70) $$\begin{array}{c} U^{\prime }=-\mu \frac{{\left(S-S^{*}\right)}^{2}}{S}+B_{2}\left(1-l\right)\beta S^{*}I^{*}\left(2-\frac{1}{x}-x\right)+B_{1}l\beta S^{*}I^{*}\left(2-\frac{1}{x}-\frac{xz}{y}-\frac{y}{z}+1\right)=-\mu \frac{{\left(S-S^{*}\right)}^{2}}{S}+B_{2}\left(1-l\right)\beta S^{*}I^{*}\left(2-x-\frac{1}{x}\right)+B_{1}l\beta S^{*}I^{*}\left(3-\frac{1}{x}-\frac{y}{z}-\frac{xz}{y}\right). \end{array}$$

By the arithmetic mean-geometric mean inequality, for equality, if and only if*S* = *S*^∗^and*y* = *z* = *u*, the last expression must be less than or equal to zero. Thus, we have *U*′ ≤ 0 with equality if and only if *S* = *S*^∗^ and *L*/*L*^∗^ = *I*/*I*^∗^ = *R*/*R*^∗^. By LaSalle's Invariance Principle [36], for each solution, the omega-limit set remains in an invariant set that is contained in *Ω* = {(*S*, *L*, *I*, *R*): *S* = *S*^∗^, *L*/*L*^∗^ = *I*/*I*^∗^ = R/*R*^∗^}. Since *S* must be in *S*^∗^, *S*′ turns zero, which implies that *I* = *I*^∗^, *L* = *L*^∗^, and *R* = *R*^∗^. Thus, there is only invariant set in *Ω* which is singleton {*E*_1_}. For each solution that intersects, ℝ_+0_^4^{*L* = *I* = *R* = 0} limits to *E*_1_, which concludes that the disease persistence equilibrium *E*^∗^ of (1) is globally asymptotically stable in ℝ_+0_^4^{*L* = *I* = *R* = 0} [24].

**Lemma 2 .**

The infectious persistence equilibrium (*E*^∗^) of the model (1) is globally asymptotically stable when *ℛ*_0_ > 1, and the disease persists in the populations for a long time.

## 7. Parameter Estimation

In this section, we obtain the value of the unknown parameters for the model (1). To estimate parameter values, we have assumed the initial condition of the state variables as (*S*_0_, *L*_0_, *I*_0_, *R*_0_) = (10000, 0, 1, 0). There are seven parameters in our model which are to be obtained. Among these parameters, natural mortality rate*μ*is estimated as 0.002; the recruitment of susceptible class*λ* = *μS*_0_ = 20; the rate which leaves*L*(*t*)for*I*(*t*), i.e., incubation period*δ* = 1/7; and the fraction of*S*(*t*)which moves to*L*(*t*);*l* = 0.95; and disease-induced mortality rate is estimated as*α* = 0.0054. These are derived from the data in the literature [30]. And the rest of the parameters are disease transmission rate *β* and the recovered rate *γ* which have to be fitted; therefore, *θ* = (*β*, *γ*). Consider the initial value of the parameters to be *ω*_0_ = (*λ*, *μ*, *α*, *l*, *β*, *δ*, *γ*) = (20,0.002,0.0054,0.95,0.0000065, 1/7, 0.005), and the initial condition of the state variables is (*S*_0_, *L*_0_, *I*_0_, *R*_0_) = (10000, 0, 1, 0). Using the initial value of the parameters and the initial conditions of the state variables, the value of the unknown parameters is fitted to the model (1) with the help of the nonlinear least square (NLS) method.  Table 1 contains the description and estimated or the best fitted values of the parameters. Here, we have simulated the cumulative value of the daily case data, which are illustrated in Figures 2 and 3 that also represent the population dynamic of the susceptible, latent, and infected population *S*(*t*), *L*(*t*), and *I*(*t*), respectively. From these figures, it is observed that the infected population (*I*-class) increases significantly upon the infection and arrives at the peak at the 36th day (*I*(43) = 3.126 × 10^3^); after that, it is decaying.

## 8. Numerical Results

To further investigate the behaviour of the model (1), we conducted various numerical investigations applying the estimations that are gained and given in Table 1. For this intention, we consider two parameter sets resembling the cases of stability of the infectious persistence equilibrium, where *ℛ*_0_ > 1, and disease extinction steady state, where *ℛ*_0_ < 1. The outcomes obtained for both equilibria with stability analysis are also numerically demonstrated using MATLAB R2018a.

Using the parameter values from Table 1, the basic reproductive ratio becomes *ℛ*_0_ = 5.86 > 1 thereby signifying the asymptotic stability of the infected steady state. For this reason, different initial conditions of (*S*_0_, *L*_0_, *I*_0_, *R*_0_) are chosen as IC1 = (10000, 0, 1, 0), IC2 = (8000, 0, 2, 0), and IC3 = (12000, 0, 3, 0).

Figure 4 illustrates the system dynamics of the susceptible, latent, and infected population for the three initial conditions within two years, i.e., 730 days. In Figure 4(a), the susceptible population decays very sharply and reaches the nadir at 189, 283, and 134 for IC1, IC2, and IC3, respectively. As time increases, they are again increasing together and reaching a peak point of approximately 2782. Again, it is decreasing and reaches another nadir at 1525. Further, it is increasing and asymptotically stable at 1706 within two years; i.e., susceptible population would be constant. In Figure 4(b), the latent population increases sharply and reaches the first peak points 3136, 2200, and 4161 for IC1, IC2, and IC3, respectively; then, they are decreasing sharply and reach a nadir at 5 together within 3.67 months and stable about three months. As time increases, they are again increasing and reach the second peak at 305 within the next 3 months. Again, they are decaying and reach another nadir at 51 within the next 3.67 months. Further, they increase and reach the third peak point of 158 within the next 4 months. They are decaying further and reach another nadir at 85 within the next 4 months. As time increases, they are increasing further and asymptotically stable at 109 within 2 years. Moreover, in Figure 4(c), the infected population increases very sharply and reaches the first peak points at 2383, 1739, and 3058 for the same initial conditions; then, they are decaying as they are increased and reach a nadir at 5 together within 4 months and stable about three months. As time increases, they are again increasing and reaches the second peak at 280 within the next 3.33 months. Again, they are decaying and reach another nadir at 47 within the next 3.67 months. Further, they are increasing and reach the third peak at 145 within the next 4 months. They are decaying further and reach another nadir at 80 within the next 3.67 months. As time increases, they are increasing further and asymptotically stable at 100 within 2 years.

Figure 5 illustrates the system's phase portrait for different initial conditions. It represents the relative change of the susceptible *S*(*t*), latent *L*(*t*), and infected populations *I*(*t*) to one another over time by a single trajectory. It also characterises the stability of the system. For different initial conditions, the trajectories are approaching a single point which specifies the disease persistence equilibrium point *E*^∗^ = (1706,109,100,7814) when the basic reproduction number *ℛ*_0_ = 5.86 > 1. In this case, the trajectories approach the long-term steady state, and the disease persists in the populations for *t*⟶∞.

For disease-extinction equilibrium, we assume the value of infection transmission rate *β* different from Table 1 as *β* = 0.000005. Therefore, the basic reproductive ratio is evaluated as *ℛ*_0_ = 0.302 < 1. For this case, the disease dynamics are illustrated in Figure 6 for the same initial conditions. The latent and infected populations are converged to 0 within 4 months that are illustrated in Figures 6(b) and 6(c), respectively, which indicates that the disease will be extincted from the populations by itself within 120 days. However, in Figure 6(a), in the susceptible population, only positive values remain for the different initial conditions that indicate the infection-free steady state. Moreover, Figure 7 illustrates the infection-free steady states and the interaction between the populations by three trajectories for three different initial conditions. The trajectories are approaching a single point defined as infection-free steady-state *E*^0^ = (10000, 0, 0, 0) and remain at this point for *t*⟶∞.

## 9. Conclusion

We have proposed a diphtheria epidemic model and found two steady-state equilibrium points: one is disease extinction equilibrium point *E*^0^ (37), and another is infectious persistence equilibrium point *E*^∗^ (38). We have formulated the basic reproductive number in terms of parameters. We have also shown analytically that the infectious extinction equilibrium (37) is globally asymptotically stable when the basic reproductive ratio *ℛ*_0_ does not exceed unity; the infection is dispelled by itself from the populations. The infectious persistence equilibrium (38) is also globally asymptotically stable when the basic reproductive ratio *ℛ*_0_ is more than unity; the disease persists in the populations at a certain level. We have fitted the daily case data from November 8, 2017, to December 27, 2017, given in [30] to our model and have evaluated the parameter's value. Both equilibria have been analyzed numerically and found a lot that matches the real scenario. We have found the first peak at 38 days for IC1 that matches with the real data, and the second and third peaks have been found at 310 days and 1.5 years, respectively, which also a lot matches with the real scenario, like the highest infection found after one month, given in [30, 41–44]. The enumerated infectious persistence equilibrium *E*^∗^ is (1706,109,100,7814) and infection-free steady-state *E*^0^ is (10000, 0, 0, 0). A statistical model was used to calculate the numeric value of the basic reproductive ratio *ℛ*_0_ in [30] and deduced a range of estimates ranging from 4.7 to 14.8 with a median estimate of 7.2. But in this study, it has calculated *ℛ*_0_ = 5.86 by involving a mathematical model, which indicates that the infection rate is very high. This study suggests applying treatments to control the diphtheria epidemic. Lastly, we hope that this study will be focused on the assumption of control strategies by constituents and policymakers.

## Figures and Tables

**Figure 1:** Diagram interaction of each compartment.

**Figure 2:** The diphtheria model (1) simulation in log scale.

**Figure 3:** The fitted diphtheria model (1).

**Figure 4:** Population dynamics interaction between *S*(*t*), *L*(*t*), and *I*(*t*) of diphtheria model (1) when *ℛ*_0_ = 5.86 > 1 for different initial conditions.

**Figure 5:** System's phase portrait of diphtheria model (1) in 2D and 3D when *ℛ*_0_ = 5.86 > 1 for different initial conditions.

**Figure 6:** Population dynamics interaction between *S*(*t*), *L*(*t*), and *I*(*t*) of diphtheria model (1) when *ℛ*_0_ = 0.302 < 1 for different initial conditions.

**Figure 7:** System's phase of diphtheria model (1) in 3D when *ℛ*_0_ = 0.302 < 1 for different initial conditions.

**Table 1:** Description and value of the parameters of the diphtheria model.

Parameter	Description	Value	Source
*λ*	The recruitment of susceptible class	200 persons day^−1^	Estimated
*μ*	Natural mortality rate	0.002 day^−1^	Estimated
*α*	Disease induced mortality rate	0.0054 day^−1^	Estimated
*β*	Disease transmission rate	0.000097 persons^−1^ day^−1^	Fitted
*l*	The fraction of *S*(*t*) which moves to *L*(*t*)	0.95	Estimated
*γ*	Recovered rate	0.156 day^−1^	Fitted
*δ*	The rate which leaves *L*(*t*) for *I*(*t*)	0.143 day^−1^	Estimated

## Data Availability

The data supporting the study are accessed from the study “R. Matsuyama, A. R. Akhmetzhanov, A. Endo, H. Lee, T. Yamaguchi, S. Tsuzuki, H. Nishiura, Uncertainty and sensitivity analysis of the basic reproductive number of the diphtheria: a case study of a Rohingya refugee camp in Bangladesh, November-December 2017, PeerJ, 6 (2018) 4582. doi:10.7717/peerj.4583.”
